The article "Large intergenic non-coding RNA-ROR reverses gemcitabine-induced autophagy and apoptosis in breast cancer cells" was retracted in 2025. Reasons: plagiarized images; duplicated images; overlap with other authors' work.

# Large intergenic non-coding RNA-ROR reverses gemcitabine-induced autophagy and apoptosis in breast cancer cells

**DOI:** 10.18632/oncotarget.10730

**Published:** 2016-07-20

**Authors:** Yao-Min Chen, Yu Liu, Hai-Yan Wei, Ke-Zhen Lv, Pei-Fen Fu

**Affiliations:** ^1^ Department of Breast Surgery, The First Affiliated Hospital of Zhejiang University, Hangzhou 310000, P.R. China

**Keywords:** breast cancer, linc-ROR, gemcitabine, large intergenic non-coding

## Abstract

The purpose of this study was to elucidate the potential role of long intergenic non-protein coding RNA, regulator of reprogramming (linc-ROR) in gemcitabine (Gem)-induced autophagy and apoptosis in breast cancer cells. MDA-MB-231 cells were treated with short hairpin RNA (shRNA) to knockdown *Linc-ROR* expression in the presence of Gem. Gem treatment alone decreased cell survival and increased both apoptosis and autophagy. Gem treatment also increased the expression of LC3-II, Beclin 1, NOTCH1 and Bcl-2, but decreased expression of p62 and p53. Untreated MDA-MB-231 cell lines strongly expressed linc-ROR, but *linc-ROR* knockdown decreased cell viability and expression of p62 and p53 while increasing apoptosis. *Linc-ROR* knockdown also increased LC3-II/β-actin, Beclin 1, NOTCH1, and Bcl-2 expression, as well as the number of autophagic vesicles in MDA-MB-231 cells. Linc-ROR negatively regulated *miR-34a* expression by inhibiting histone H3 acetylation in the *miR-34a* promoter. We conclude that linc-ROR suppresses Gem-induced autophagy and apoptosis in breast cancer cells by silencing *miR-34a* expression.

## INTRODUCTION

In women, breast cancer is the most prevalent form of cancer, and is second only to lung cancer as the cause of cancer-related death [1, 2]. Family history, genetic susceptibility, and environmental risk factors all contribute to the prevalence of this disease [3–5]. Neoadjuvant chemotherapy has become a reasonable treatment, among which bevacizumab, capecitabine, gemcitabine (Gem) and taxanes have been shown to improve outcomes in patients with metastatic breast cancer [6]. Gem is a nucleoside analog, and is widely used in various carcinomas, including non-small cell lung cancer, pancreatic cancer, bladder cancer, and breast cancer [7–10]. Gem regulates the VMP1-mediated autophagy pathway and increases apoptosis in tumors [11, 12]. The regulation of autophagy and apoptosis by Gem is reflected by increased expression of autophagy- (Beclin1, ATG16L1, LC3) and apoptosis-related proteins (Bcl-2, Bax) [12–15].

Large intergenic non-coding RNAs (lincRNAs) are RNAs contained within intergenic regions identified by histone lysine 4 and lysine 36 chromatin marks [16]. Mutations in lincRNA genes are associated with many human diseases [17–19]. LincRNAs have crucial roles in controlling gene expression during cell development and differentiation, and are important for chromosomal dosage compensation, genomic imprinting, cell differentiation, and organogenesis [20]. *LincRNAs, regulator of reprogramming (linc-RoR)* located at chromosome 18q21.31 and consisted of 4 exons, with a length of 2.6 kb, and was important in the regulation of reprogramming process of cells [21]. The linc-RoR is highly expressed in malignant liver cancer cells [22], and silencing of linc-ROR represses breast cancer cell growth and lung metastasis *in vivo* [23]. Hou et al have found that ROR was higher in breast cancer tissues and could promote occurrence and metastasis of breast cancer through regulating epithelial to mesenchymal transition [23]. Previous studies also showed that lincRNAs could influence the expression of genes by regulating the shear process of mRNA, such as Linc-ROR binding with miR-145 regulating cell differentiation and cancer progression [23, 24].

Autophagy is a vital process that degrades damaged cellular components and mediates their recycling, while apoptosis is a fundamental process that regulates tissue homeostasis [25]. Although linc-ROR is upregulated in triple-negative breast cancer [26], very little is known about the role of linc-ROR in autophagy and apoptosis. MiR-34a, located on chromosome 1p36.23, is a member of the miR-34 family, and it may target several apoptosis inhibitor genes to induce apoptosis, which has a close relation to its regulation of autophagy [27, 28]. It has been demonstrated that the miR-34a expression was altered in various cancers, including breast cancer, lung cancer, and prostate cancer [29, 30]. Moreover, it has also been reported that p53-inducible *miR-34a* participates in cell cycle arrest, senescence, and apoptosis by down-regulating the expression of Bcl-2 and promoting expression of b-Myb, a protein involved in cell cycle progression [31–33]. Therefore, we hypothesized that linc-ROR participates in autophagy and apoptosis in breast cancer by regulating the expression of *miR-34a*.

## RESULTS

### Gem decreases MDA-MB-231 cell viability

A CCK-8 assay was used to measure MDA-MB-231 cell viability after treatment with different concentrations of Gem. Gem inhibited cell viability in a dose-dependent manner (Figure 1). The IC_50_ of Gem in MDA-MB-231 cells at 24 h was 0.05 ± 0.018 μmol/ml, therefore a Gem concentration of 0.05 μmol/ml was used for subsequent experiments.

**Figure 1:** Gem treatment reduces cell viability and induces apoptosis in MDA-MB-231 cells CCK8 was applied to detect cell viability after cells were treated with Gem for 24h, 48h, and 72h. Experiments were independently conducted three times; Gem, gemcitabine.

### Autophagosome assembly and autophagy-related protein expression after Gem treatment

Inverted fluorescence microscope revealed that MDC-positive cells presented with bright blue spots. As seen in Figure 2A, Gem-treated MDA-MB-231 cells had increased numbers of blue spots compared with the blank treatment group. Gem-treated MDA-MB-231 cells visualized by TEM had many autophagic vacuoles, which included organelles in various phases of degradation. No such autophagic vacuoles were observed in the blank treatment group (Figure 2B).

**Figure 2:** Gem treatment increases autophagosome- and autophagy-related protein expression in MDA-MB-231 cells **A.** MDA-MB-231 cells were under Gem or negative treatrment for 48h, followed by 50 μmol/L of MDC treatemnt for 15 min. Cell staining was observed by an inverted fluorescence microscope; **B.** MDA-MB-231 cells were under Gem treatment or negative treatrment for 48h. Ultrastructure was examined using TEM. White arrow, classical autolysosome with double membrane containing organelles in various phases of degradation; black arrow, matured lysosomes; **C-E.** MDA-MB-231 cells were treated with 0.05 μmol/ml of Gem for 48h. Western blot was used to observe the transformation of LC3-I (18KDa) and LC3-II (16 KDa) and expression of p62, Beclin 1, and NOTCH1; **F.** MDA-MB-231 cells were transiently transfected with EGFP-LC3 plasma and then treated with 0.05 μmol/ml of Gem for 48h. Confocal microscopy was used to locate fluorescence. Bright green spots represent the autophagosome. LC3-II+ bright green spots in more than 75 cells were calculated. Comparisons between the control group and other treatment groups were assessed; *, *P* < 0.05; **, *P* < 0.01, ***, *P* < 0.001

Western blot was performed to detect the expression of LC3, p62, Beclin 1 and NOTCH1 in Gem-treated MDA-MB-231 cells. The LC3-II/b-actin ratio was used as an index of autophagy since LC3-I had unstable expression, while LC3-II was rather stable. Gem-treated cells had an elevated LC3-II/b-actin ratio (Figure 2C) and increased expression of Beclin 1 and NOTCH1, but decreased p62 expression (Figure 2D) in comparison to the blank treatment group (all *P*<0.05; Figure 2E). To further elucidate whether Gem treatment induces autophagy, we transiently transfected EGFP-LC3 plasma in MDA-MB-231 cells. Once autophagy occurred, the fluorescence in cells was relocated in the cytoplasm and detected as bright green fluorescent spots. Gem treatment for 48h increased the number of bright green fluorescence spots in comparison with the blank treatment group, suggesting that Gem increases autophagy in MDA-MB-231 cells (Figure 2F).

### Apoptosis rate and expression of apoptosis-related proteins after Gem treatment

Flow cytometry was used to observe apoptosis in MDA-MB-231 cells after treatment with Gem for 48h. Compared with the blank treatment group, Gem-treated cells had increased rates of apoptosis (all *P*<0.05; Figure 3A). The protein p53 promotes apoptosis, while Bcl-2 inhibits apoptotic progression. Western blots showed that Gem increased p53 expression but reduced Bcl-2 expression, when compared to the blank group (all *P*<0.05; Figure 3B, C).

**Figure 3:** Gem induced apoptosis in human breast cancer MDA-MB-231 cells **A.** Apoptosis rate of MDA-MB-231 cells detected by flow cytometry after 0.05 μmol/ml of Gem was added for 48h. Scatter plot and analysis of cell apoptosis; **B.** Detection of protein using Western blot. **C.** Relative expression of Bcl-2 and p53, presented as mean ± SE. Experiments were independently conducted three times; *,*P* < 0.05; Gem, gemcitabine.

### *Linc-ROR* silencing decreases cell viability and induces apoptosis in Gem-treated MDA-MB-231 cells

RT-PCR revealed that, compared with human MCF10A cells, MDA-MB-231 cells had elevated expression of *linc-ROR* (*P* < 0.001; Figure 4). ROR silencing decreased the expression of *linc-ROR* (*P*<0.05, Figure 5A). The blank treatment group had the highest cell viability at 24h, 48h and 72h, followed by the sh-Ctrl+Gem group, the Gem group, and the sh-ROR+Gem group, respectively. Pair-wise comparisons on cell viability were statistically significant (all *P*<0.05) except between the sh-Ctrl+Gem group and Gem group (Figure 5B). Flow cytometry indicated that the blank group had the lowest apoptotic rate, followed by the sh-Ctrl+Gem group, and the Gem group, while the sh-ROR+Gem group had the highest apoptotic rate. Pair-wise comparisons on apoptotic rate were statistically significant (all *P*<0.05) except between the sh-Ctrl+Gem group and the Gem group (Figure 5C). These results suggested that *Linc-ROR* silencing decreases cell viability and increases the rate of apoptosis in Gem-treated MDA-MB-231 cells.

**Figure 4:** Linc-ROR expression in MDA-MB-231 and MCF10A cells by reverse transcription polymerase chain reaction (RT-PCR)

**Figure 5:** Linc-ROR influences cell viability and apoptosis in Gem-treated MDA-MB-231 cells **A.** *linc-ROR* expression in ROR-shRNA transfected MDA-MB-231 cells by qRT-PCR; **B.** Cell viability detected by CCK8 assay; **C.** Apoptosis rate detected by flow cytometry; qRT-PCR, quantitative reverse transcription polymerase chain reaction; *, *P* < 0.05; Gem, gemcitabine.

### *Linc-ROR* knockdown promotes the expression of autophagy- and apoptosis-related proteins in Gem-treated MDA-MB-231 cells

Western blots revealed that the sh-ROR+Gem group had the highest LC3-II/b-actin ratio, as well as expression of Beclin 1, NOTCH1 and p53. The next highest was the sh-Ctrl+Gem group, followed by the Gem group and the blank group, respectively. The sh-ROR+Gem group had the lowest expression of p62 and Bcl-2, followed by the sh-Ctrl+Gem group, the Gem group, and the blank group, respectively. Pair-wise comparisons showed statistical significance (all *P*<0.05) except between the sh-Ctrl+Gem group and the Gem group (Figure 6). These results suggested that *linc-ROR* silencing promoted the expression of autophagy-related proteins (LC3-II, Beclin 1, NOTCH1) and the pro-apoptotic protein, p53, but decreased the expression of the autophagy protein, p62, and the anti-apoptotic protein, Bcl-2.

**Figure 6:** Linc-ROR influences expression of apoptosis and autophagy related proteins in Gem-treated MDA-MB-231 cells **A.** Detection of protein using Western blot; **B.** Transformation between Lc3-I (18KDa) and LC3-II (16 KDa) in MDA-MB-23 cells using Western blot; **C.** Expression of apoptosis- and autophagy-related proteins in Gem-treated MDA-MB-231 cells using Western blot; *, *P* < 0.05.

### *Linc-ROR* silencing promotes autophagosome assembly in Gem-treated MDA-MB-231 cells

Confocal microscopy showed that MDC-positive cells in all treatment groups had bright blue fluorescence spots. The strongest fluorescence was found in the sh-ROR+Gem group, followed by the sh-Ctrl+Gem group, the Gem group and the blank group, respectively (Figure 7A). TEM imaging revealed that the sh-ROR+Gem group had more autophagic vacuoles when compared with the Gem group, while both the sh-Ctrl+Gem group and the Gem group had elevated autophagic vacuole numbers in comparison to the blank group (Figure 7B). All pair-wise comparisons among the four groups were significant (all *P*<0.05) except for between the sh-Ctrl+Gem group and the Gem group. These results implied that *linc-ROR* silencing increases the number of autophagic vacuoles in Gem-treated MDA-MB-231 cells.

**Figure 7:** Linc-ROR influences autophagosome assembly in Gem-treated MDA-MB-231 cells **A.** Staining of MDA-MB-231 cells visualized by inverted fluorescence microscope; **B.** Ultrastructure in MDA-MB-231 cells by TEM. White arrow, classical autolysosome with double membrane containing organelles in various phases of degradation; black arrow, matured lysosomes; Gem, gemcitabine.

### *Linc-ROR* influences cell apoptosis and autophagy by inhibiting *miR-34a*

The target gene of NOTCH1, *miR-34a*, is involved in regulating apoptosis and autophagy in breast cancer [36, 37]. Our *in silico* analysis revealed that linc-ROR has miRNA binding sites including for miR-34a (Figure 8A, B); therefore, we hypothesized that linc-ROR may interact with miR-34a to induce autophagy. qRT-PCR was conducted to detect expression of *miR-34a* in the four cell treatment groups. Expression of *miR-34a* was highest in the sh-ROR+Gem group compared with the other three groups (all *P*<0.05). The sh-ROR+Gem group and the sh-Ctrl+Gem group had elevated *miR-34a* expression when compared with blank group (both *P*<0.05), while no difference was detected between the sh-ROR+Gem group and the sh-Ctrl+Gem group (*P*>0.05) (Figure 8C), suggesting that linc-ROR may negatively regulate *miR-34a* expression. Western blots demonstrated that, compared with the sh-ROR+Vector group, expression of NOTCH1 and p53 were decreased while expression of p62 and Bcl-2 were increased in the sh-ROR+Gem+inhibitors group (all *P* < 0.05) (Figure 8D-F).

**Figure 8:** Linc-ROR negatively regulates *miR-34a* **A.** Wild-type and mutated reporter constructs of Notch1 3′UTR; **B.** Analysis of the binding site between linc-ROR and miR-34a; **C.** Detection of linc-ROR expression by RT-PCR; **D.** Detection of protein using Western blot; **E.** Transformation between Lc3-I (18KDa) and LC3-II (16 KDa) in MDA-MB-23 cells using Western blot; **F.** Expression of apoptosis- and autophagy-related proteins by Western blot; *, *P* < 0.05; RT-PCR, reverse transcription polymerase chain reaction.

### linc-ROR regulation of *miR-34a*

ChIP was used to observe acetylation of histone H3 in the *miR-34a* promoter [24] Compared with the sh-ROR+Gem group, *miR-34a* promoter H3 acetylation was decreased in the Gem group, which was consistent with the findings of *miR-34a* expression (Figure 9). Our results suggested that *linc-ROR* silencing inhibited acetylation of histone H3 in the miR-34a promoter and reduced *miR-34a* expression. Decreased expression of *miR-34a* could then inhibit Gem-induced apoptosis and autophagy in breast cancer cells.

**Figure 9:** Acetylation of histone H3 in the *miR-34a* promoter in the Gem-treated group and the sh-ROR+Gem group Gem, gemcitabine; *, *P* < 0.05.

## DISCUSSION

In this study, we carried out a comprehensive exploration of the possible role of linc-ROR in Gem-induced apoptosis and autophagy in breast cancer cells. Our results confirmed the inhibitory role of Gem on apoptosis and autophagy in a human breast cancer (MDA-MB-231) cell line. We also found evidence that *linc-ROR* silencing may result in suppression of cell viability and promotion of apoptosis and autophagy, thus contributing to the control of breast cancer progression and development. To further clarify the mechanism of *linc-ROR* reversal of Gem inhibition of apoptosis and autophagy, we conducted a miRNA analysis and found that linc-ROR may inhibit the expression of *miR-34a* by suppressing acetylation of histone H3 in the *miR-34a* promoter. Programmed cell death, one of the most important regulatory cellular processes, comes in two forms: apoptosis and autophagy [38]. Apoptosis is indicated by cell shrinkage, membrane blebbing, and phagocyte release into apoptotic bodies. In contrast, autophagy is detected by the presence of autophagosomes, the autolysosome, and an intact nucleus in the cell [39]. In our study, CCK8 assays, flow cytometry, and Western blots all showed that Gem treatment reduced cell viability and increased autophagy and apoptosis in breast cancer (MDA-MB-231) cells. Changes in autophagy and apoptosis were reflected by the presence of autophagic vacuoles, in addition to expression of autophagy-related proteins (LC3, p62, Beclin 1 and NOTCH1) and apoptosis-related proteins (Bcl-2, p53).

Autophagy is a process of cell growth control, and decreased expression of autophagy proteins may contribute to the development and/or progression of human malignancies [40]. In pancreatic cancer, Gem has been a commonly used cancer therapy with a response rate of approximately 20% that triggers autophagy by a reactive oxygen species (ROS)-mediated mechanism [41]. The regulation of autophagy pathways by ROS may interact with each other pathways in disease progression and therapeutic response [42]. Whether a cell lives or dies is largely determined by interactions among members of the Bcl2 protein family [43]. In addition, cancer, ischemia, cholestasis, and atherosclerosis are all closely associated with deregulated levels of apoptosis in which p53 dysfunction has a prominent role [44]. Chen et al have found that overexpressed linc-ROR may decrease the sensibility of 5-FU and paclitaxel with decreased E-cadherin expression, N-cadherin expression, and invasion ability, which may be an important marker for multidrug resistance of breast cancer, and the linc-ROR up-regulation was important for chemotherapy tolerance and invasion of breast cancer [45]. In our study, the Gem-treated MDA-MB-231 cells had decreased Bcl-2 expression and increased p53 expression, suggesting that Gem could promote apoptosis in breast cancer.

Our study also verified that linc-ROR was highly expressed in human breast cancer MDA-MB-231 cells. Moreover, linc-ROR silencing decreased cell viability and elevated rates of apoptosis and autophagy. Results from our ChIP experiment suggested that linc-ROR may negatively regulate miR-34a in MDA-MB-231 cells. Therefore, we hypothesized that linc-ROR inhibits Gem-induced apoptosis and autophagy by suppressing acetylation of histone H3 in the miR-34a promoter, thereby reducing miR-34a expression. Linc-ROR was first identified as a promoter of reprogramming of human induced pluripotent stem cells (iPSCs), and it was reported to have a key role in the maintenance of iPSCs and embryonic stem cells (ESCs) by preventing the activation of cellular stress pathways, including the p53 response [46, 47]. Highly expression of linc-ROR was found in ESCs and iPSCs, which is resulted by the regulation of linc-RoR by pluripotency transcription factors, for example, Oct4, Sox2 and Nanog [48]. Previous studies unveiled that linc-ROR could act as a p53 repressor in response to DNA damage, and the knockdown of linc-RoR leads to a modest increase in apoptosis and activation of p53 pathways [20, 49], which may contribute to breast cancer tumourigenesis and metastasis. *p53* is a tumor suppresser gene that induces apoptosis in a large number of human malignancies [50]. p53 participates in the cellular response to genotoxic stress by targeting downstream miRNAs, and miR-34a participates in the apoptotic program triggered by p53 activation [32]. In addition, siRNA to linc-RoR increased the activity of p53, suggesting that the effects of linc-ROR are mediated through p53-dependent signaling [51]. Moreover, miR-34a directly inhibits the expression of Bcl-2 and exerts its tumor suppressive effects, including cell proliferation inhibition, cell cycle arrest, and induction of apoptosis [52]. These results further enhance our conclusions that linc-ROR may repress Gem-induced apoptosis by regulating miR-34a.

In terms of autophagy, our results showed that *linc-ROR* silencing promoted the expression of autophagy related proteins (LC3-II, Beclin 1, NOTCH1) and decreased p62 expression. miR-34a synthetic mimics trigger growth inhibition and apoptosis in multiple myeloma cells by down-regulating canonical targets, Bcl-2, CDK6, and NOTCH1, both *in vitro* and *in vivo* [53]. In addition, Li et al have aslo demonstrated that miR-34a negatively correlated with the mRNA and protein expression levels of Notch1, and the overexpression of miR-34a may sensitize MCF-7/ADR cells to adriamycin [36]. In agreement with our results, over-expression of miR-34a reduces the expression of ATG4B, Beclin-1, and LC3B II/I in prostate cancer cells by downregulating p-AMPK and upregulating p-Mtor, an essential pathway related to cellular autophagy [54, 55].

In summary, we provide strong evidence that linc-ROR inhibits Gem-induced apoptosis and autophagy by decreasing *miR-34a* expression. Our findings may contribute to the development of a new therapeutic strategy to improve breast cancer treatment outcomes. However, further studies are required to examine the modulation of Gem-induced autophagy and apoptosis in breast cancer cells by linc-ROR.

## MATERIALS AND METHODS

### Cell culture

Human breast cancer cells (MDA-MB-231) and human immortalized mammary epithelial cells (MCF10A) were purchased from ATCC. MCF10A cells were cultured in an incubator (37°C, 5% CO_2_) using Dulbecco's modified Eagle's medium (DMEM)-F12 (Gibco Company, USA) medium containing 5% horse serum 20 ng/ml epidermal growth factor (EGF; Peprotech Company, USA), 0.5 mg/ml hydrocortisone (Gibco Company, USA), 100 ng/ml choleratoxin (Gibco Company, USA), 10 mg/ml insulin and antibiotics (Gibco Company, USA), while MDA-MB-231 cells were cultured in L-15 medium containing 10% fetal bovine serum (FBS; Gibco Company, USA) and incubated at 37°C without CO_2_.

### Cell groupings and transfection

(1) MDA-MB-231 cells were treated with different concentrations of Gem, with a blank group remaining untreated for comparison.
(2) MDA-MB-231 cells were classified into four groups: a) sh-ROR+Gem group (treated with 0.05 μmol/ml of Gem [Sigma-Aldrich Company, USA] for 24h, followed by sh-ROR transfection), b) sh-Ctrl+Gem group (treated with 0.05 μmol/ml of Gem for 24h, followed by negative control of sh-ROR transfection), c) Gem group (treated with 0.05 μmol/ml of Gem for 48h) and d) blank group (no treatment applied). According to instructions of the transfection reagents (Invitrogen Company, USA), MDA-MB-231 cells were seeded in 6-well plates 24h before transfection. Culture medium was replaced with 2 ml DMEM 1h before the transfection was conducted. The transfection complex included sh-ROR (silencing expression of linc-ROR) and sh-Ctrl (negative control). The primer sequences for sh-Ctrl and sh-ROR were: GATCCCCTTCTCCGAACGTGTCACGTTTCAAGAGAACGTGACACGTTCGGAGAATTTTTC and GATCCCCCCTGAGAGTTGGCATGAATTTCAAGAGAATTCATGCCAACTCTCAGGTTTTTC, respectively. All sequences were synthesized by Sangon (Shanghai, China). The DMEM medium in each well was removed and replaced with 200 μl of opti-MEM and 800 μl transfection mixture. The plates were incubated at 37°C for 4h, after which 500 μl of DMEM containing 3X FBS was added, followed by incubation at 37°C for another 24h. Subsequently, cells were collected and total protein was extracted for further analysis.
(3) MDA-MB-231 cells were grouped into the following groups: a) sh-ROR+Gem+inhibitors group (treated with 0.05 μmol/ml of Gem for 24h and then co-transfected with sh-ROR and miR-34a inhibitor), b) sh-ROR+Gem+NC group (treated with 0.05 μmol/ml of Gem for 24h and then transfected with sh-ROR and negative control of miR-34a inhibitor) and c) sh-ROR+Gem group (treated with 0.05 μmol/ml of Gem for 24h and then transfected with sh-ROR). One day before transfection, MDA-MB-231 cells at logarithmic growth phase were sub-cultured in 6-well plates overnight with DMEM containing 10% FBS. Transfection was conducted after cell fusion reached 30%~50%. DMEM free from serum or antibiotic was added to dilute the transfection mixture (50 pmol). Transfection mixtures were then mixed with Lipofectamine 2000 (Invitrogen Company, USA). After maintaining the mixtures at room temperature for 20 min, they were added to the cells, followed by incubation for 5h (37°C, 5% CO_2_). The medium was replaced by and cells were further incubated for 24h.

### GFP-LC3 observation

GFP-LC3 plasma (constructed by our laboratory) was transiently transfected into human breast cancer MDA-MB-231 cells followed by treatment with Gem (0.05μg/ml) for 48h. A blank group (no treatment) was used as a control. Green GFP-LC3 cells were observed under a fluorescence microscope (× 400) (Olympus Company, Japan), with 300 cells randomly selected and photographed for each group. Experiments were repeated three times and mean values were obtained.

### Cell Counting Kit-8 (CCK-8) assay

MDA-MB-231 cells in the logarithmic growth phase were selected and rinsed twice in PBS. Then cells were trypsinized and made into single-cell suspension using a pipette. Cells numbers were calculated. Cells (5 × 10^3^) were plated in 96-well plates with 200 μL volume in each well and incubated at 37°C with 5%CO_2_. Cell adherence was observed the next day and then the initial culture medium discarded. Gem was added to the treated cell groups, while the control group received DMEM of the same volume. Cells were incubated for another 24h and 20 μL of CCK8 (Sigma Company, USA) was added in a 96-well plate. Plates were then incubated for 3h at 37°C with 5% CO_2._ The absorbance at 48h and 72h was measured with a microplate reader at a wavelength of 450nm. Measurements were repeated three times. Cell survival rate was calculated based on following formula: cell survival rate% = [1-(A_450_Sample-A_450_blank)/(A_450_Control-A_450_blank)] × 100%.

### Detection of cell apoptosis by flow cytometry

MDA-MB-231 cells in the logarithmic growth phase were selected and rinsed twice in PBS. Cells were evenly mixed with 500 μ l of pre-cooled 1X binding buffer, 5 μL of Annexin-V-FITC (eBioscience, San Diego, USA), and 2.5 μL of PI (eBioscience, San Diego, USA). Flow cytometry (BD FACSArial I cell sorter) was used to detect apoptosis. Q4 in the scatter diagram represented healthy viable cells (FITC^−^/PI^−^); Q3 represented early apoptotic cells (FITC^+^/PI^−^); and Q2 represented necrotic and late apoptotic cells (FITC^+^/PI^+^). The apoptosis rate was calculated based on following equation: apoptosis rate = early apoptosis rate (Q3) + late apoptosis rate (Q2).

### Detection of acid autophagy vesicles (AVO) by Monodansylcadaverine (MDC) staining

MDA-MB-231 cells in the logarithmic growth phase had medium removed when the cell density reached 80%~90% and were washed twice with PBS. 4 mL of Gem was added at a predetermined concentration and cells were incubated at 37°C with 5% CO_2._ Twenty-four hours later, the culture medium was removed and samples were washed twice with PBS. Next, 0.5mol/L MDC medium was added and samples were incubated at 37°C without any light exposure. One hour later, the medium was removed and cells were washed three times with PBS. Inverted fluorescence microscope (Olympus Company, Japan) was used for observation and photographs at 37°C with a 350 nm filter.

### Observation of autophagosome ultrastructure by transmission electron microscope

Cells in a culture dish were observed for morphological changes and were treated with different concentrations of Gem based on group classifications. Cells were digested with trypsin, centrifuged, and resuspended in 2.5% glutaraldehyde for 1h. After two, 15 minute washes in PBS, cells were fixed in 1% Osmium oxide for 1h, washed in ddH_2_O for 15 min (x2) and incubated with 4% Uranyl acetate for 30 min. After that, graded dehydration under 50%, 70%, and 90% ethyl alcohol was conducted (15 min each), followed by 100% ethyl alcohol dehydration for 20 min and 100% acetone dehydration for 20 min (×2). Samples were embedded and polymerized at 37°C for 24h, at 45°C for 24h and 60°C for 48h, followed by sample sectioning. After the addition of 4% uranyl acetate for 20 min and lead citrate for 5 min, cell samples were observed under a transmission electron microscope (TEM, 80Kv; Olympus Company, Japan).

### Quantitative real-time polymerase chain reaction (qRT- PCR)

Total RNA was extracted based on kit instructions (Promega Company, USA). An ultraviolet spectrophotometer was used to detect the OD260/280 value of the RNA and to calculate RNA concentration, after which RNA was preserved at −80°C for later use. Primers were designed using Primer 5.0 software and synthesized by Sangon Biotech (Shanghai, China; Table 1). Experiments were performed in accordance with procedures provided by the Reverse Transcription System A3500 (Promega Company, USA). The reaction conditions were: pre-denaturation at 95°C for 15 min for 1 cycle, then denaturation at 95°C for 10 s, and annealing at 59°C for 30s with extension at 95°C for 30 s for a total of 40 cycles. qRT-PCR was conducted with a total reaction volume of 25 μl containing 12.5 μl of Premix Ex Taq or SYBR Green Mix, 1 μl of Forward Primer, 1 μl of Reverse Primer, 1-4 μl of DNA template and ddH_2_O. *U6* was used as controls. A solubility curve was used to evaluate the reliability of PCR results. The average CT value (amplified power curve inflection point) was taken. Semi-quantitative analysis and calculation of relative expression of the target gene were performed using the 2^−ΔΔ^Ct method [34].

**Table 1:** Primers sequences for RT-PCR

PCR primers sequences	Forward (5′-3′)	Reverse (5′-3′)
U6	CTCGCTTCGGCAGCACA	AACGCTTCACGAATTTGCGT
linc-ROR	CCAGGACAATGAAACCAC	AGGAGCCCAAAGTAACAG
miR-34a	ACACTCCAGCTGGGTGGCAGTGTCTTAGCTG	CTCAACTGGTGTCGTGGAGTCGGCA
		ATTCAGTTGAGAACAACCA
miR-34a promotor CH-ip	GGCCAGCTGT GAGTGTTTCT	CAACGTGCAG CACTTCTAGG

RT-PCR, reverse transcription polymerase chain reaction.

### Western blot

According to the manufacture's instruction, RIPA lysis buffer (Pulitzer, Beijing, China) was applied to cells and protein concentrations calculated using the BCA method (ComWin Biotech Co.,Ltd, Beijing, China) [35]. Proteins were subjected to SDS-PAGE electrophoresis (Beyotime Biotechnology, China), transferred to PVDF membrane (Millipore Company, USA) at 250mA, and blocked in 3% BSA for 1h. The antibodies used were: primary LC3 antibody (Cell Signaling, USA, 4108), primary Notch1 antibody (Cell Signaling, USA, 3608), primary Beclin antibody (Cell Signaling, USA, 3738), primary P62 antibody (Abcam, UK, ab56416), primary p53 antibody (Santa Cruz Biotechnology, USA, sc-126), primary Bcl-2 antibody (Santa Cruz Biotechnology, USA, sc-7382), and anti β-actin antibody (Santa Cruz Biotechnology, USA, sc-130619). Antibodies were incubated at 4°C overnight. Membranes were washed with TBST (10 min ×3), horseradish peroxidase (HRP) labeled secondary antibodies (ZSGB-BIO, Beijing, China, ZB-2301) were added, and membranes were incubated at room temperature for 1h. A chemiluminescent substrate (Pulitzer, Beijing) was applied to develop films using an ImageQuant LAS 4000 mini Ultrasensitive chemiluminescence imager.

### Chromatin immunoprecipitation assay (ChIP)

Cells were obtained according to the kit instructions (Chromatin Immunoprecipitation Kit, Upstate). Chromatin was fixed using formaldehyde then, using a sonicator, sheared into fragments of 200-1000 bp and centrifuged. Supernatant was diluted by ChIP buffer solution and rinsed in protein G agar to decrease non-specificity. After that, samples were incubated with antibodies (Anti-ACH3 antibody or Normal Mouse IgG) for immunoprecipitation at 4°C overnight shaking. Bound chromatin was collected using a suspension of protein G agar, followed by washing in subsalt, high salinity, and LiC1 elution Buffer, and in TE buffer solution (2x). Protein was digested by addition of protease and the DNA was purified using spin columns. Purified DNA samples (ChIP and Input) were used as template for PCR and electrophoresed in a 2% agarose gel. PCR products were then sequenced to further clarify the results.

### Statistical analyses

Data was analyzed using SPSS 19.0 software. Measurement data were expressed as mean ± standard deviation $\left(\bar{x}\pm \text{SD}\right)$. Prior to One-Way analysis of variance (ANOVA), homogeneity of variance was tested. Pair-wise comparisons on means and multiple groups were analyzed by LSD-t. *P*<0.05 was considered statistically significant.
